The article "Mesenchymal stromal cells can be applied to red blood cells storage as a kind of cellular additive" was published in 2017. Journal: Biosci Rep.

# Mesenchymal stromal cells can be applied to red blood cells storage as a kind of cellular additive

**DOI:** 10.1042/BSR20170676

**Published:** 2017-09-19

**Authors:** Yaozhen Chen, Jing Zhang, Shunli Gu, Dandan Yin, Qunxing An, Ning An, Lihong Weng, Jing Yi, Jinmei Xu, Wen Yin, Xingbin Hu

**Affiliations:** 1 Department of Transfusion Medicine, Xijing Hospital, Xi’an 710032, China; 2 Department of Hematology, Tangdu Hospital, Xi’an 710037, China; 3 Department of Hematology and Hematopoietic Cell Transplantation, City of Hope, Duarte 91010, CA, U.S.A.

**Keywords:** CDPA-1, mesenchymal stromal cells, RBCs, storage lesion

## Abstract

During storage in blood banks, red blood cells (RBCs) undergo the mechanical and metabolic damage, which may lead to the diminished capacity to deliver oxygen. At high altitude regions, the above-mentioned damage may get worse. Thus, more attention should be paid to preserve RBCs when these components need transfer from plain to plateau regions. Recently, we found that mesenchymal stromal cells (MSCs) could rescue from anemia, and MSCs have been demonstrated in hematopoietic stem cells (HSCs) transplantation to reconstitute hematopoiesis *in vivo* by us. Considering the functions and advantages of MSCs mentioned above, we are trying to find out whether they are helpful to RBCs in storage duration at high altitudes. In the present study, we first found that mice MSCs could be preserved in citrate phosphate dextrose adenine-1 (CPDA-1) at 4 ± 2°C for 14 days, and still maintained great viability, even at plateau region. Thus, we attempted to use MSCs as an available supplement to decrease RBCs lesion during storage. We found that MSCs were helpful to support RBCs to maintain biochemical parameters and kept RBCs function well on relieving anemia in an acute hemolytic murine model. Therefore, our investigation developed a method to get a better storage of RBCs through adding MSCs, which may be applied in RBCs storage as a kind of cellular additive into preservation solution.

## Introduction

Red blood cells (RBCs), as an important component in blood, are essential for oxygen transportation [1]. RBCs transfusion has been a common treatment for much lower red cell number counts, hemoglobin (Hb) or hematocrit (Hct) in clinic [2]. RBCs are usually stored with citrate phosphate dextrose adenine-1 (CPDA-1) solutions for up to 35 days after blood collection in China, while the storage duration could be extended with conventional additive solutions (ASs), saline adenine glucose mannitol (SAGM), or other buffers in other countries [3,4]. During storage in blood banks, RBCs undergo the mechanical and metabolic damage, which may lead to the diminished capacity to deliver oxygen [5]. Unfortunately, the mentioned damage may get worse at high altitude regions.

The article "Mesenchymal stromal cells can be applied to red blood cells storage as a kind of cellular additive" was published in 2017. Journal: Biosci Rep.

Individuals from plain to plateau have significantly increased Hct and Hb levels to meet the oxygen requirement [4]. Environmental conditions such as high altitude affects blood cells’ morphology and phenotype [6]. Thus, more attention should be paid to preserve RBCs when these components need to transfer from plain to plateau region. In order to maintain the normal quality of RBCs during transfer, we are looking for an improved additive for the storage of RBCs.

Recently, we identified a kind of mesenchymal stromal progenitor in the adult mice bone marrow hematopoietic niche, which was important for hematopoietic stem cells (HSCs) maintenance and self-renewal [7]. We also found that mesenchymal stromal cells (MSCs) could rescue from anemia [8], and they have also been demonstrated in HSCs transplantation to reconstitute animal hematopoiesis *in vivo* by us [7,9]. Considering all the functions and advantages of MSCs mentioned above, we are trying to find out if they could be a new additive to preservation solution to support RBCs at higher altitudes.

In the current study, we assessed the potential of MSCs to help RBCs maintain their viability and function during storage duration in plateau area. We found that MSCs maintained a better quality of RBCs, including the number of RBCs, Hct, Hb, and the oxygen-carrying capacity in preservation period. Moreover, we confirmed MSCs helped RBCs keep a superior effectiveness of transfusion in murine anemia models. Our research developed a method to get a better storage effect for RBCs through adding a small amount of MSCs to preservation solution. Therefore, our findings suggest MSCs to be a potential additive for RBCs storage.

## Materials and methods

### Mice

C57BL/6 mice (8–12 weeks old) were used in the present study. Mice were bred and maintained under SPF conditions in the Animal Center at the Fourth Military Medical University (FMMU). All the animal experimental protocols were conducted strictly in compliance with guidelines of the Animal Care and Use Committee of FMMU.

### Isolation and storage of mouse RBCs

Two hundred microliters of blood samples were taken from the tip of the heart of each mouse by sterile operation and suspended in a clean tube containing 200 μl CPDA-1 for preservation. The blood samples were centrifuged for 5 min at 400***g*** to get RBCs. RBCs were then resuspended at 5 × 10^12^/l in CPDA-1. The plain samples were stored at 4 ± 2°C in our lab (approximately 400 meters above sea level), while the plateau ones were taken to the lab at plateau region (approximately 2800 meters above sea level) for storage at the same temperature. The transferring process was under standard blood bank conditions.

The article "Mesenchymal stromal cells can be applied to red blood cells storage as a kind of cellular additive" was published in 2017. Journal: Biosci Rep.

### Isolation of MSCs

MSCs were obtained and characterized as our previous strategy [7,8,10]. In brief, tibias and femurs of C57BL/6 mice were obtained, and muscles and connective tissues were carefully removed from the bones with surgical scissors and razor blades. After being crushed, the bone chips were washed with PBS for at least three times to get rid of the bone marrow cells and then incubated at 37°C with collagenase I (3 mg/ml; Sigma) for 1 h. The released cells were collected from digested bone chips after filtering. RBCs lysis buffer was used to remove RBCs to get MSCs mixture. MSCs were sorted from MSCs mixture to exclude CD45 positive and Ter119 positive cells, according to mouse mesenchymal progenitor enrichment kit for compact bone (Stem Cell, catalog#19771). MSCs were identified by PE anti-mouse CD44 (IM7, BD, U.S.A.), PE anti-mouse CD51 (RMV-7, eBioscience, San Diego, U.S.A.), APC anti-mouse CD90 (OX-7, BD, U.S.A.), APC anti-mouse CD105 (MJ7/18, BioLegend, California, U.S.A.), APC anti-mouse CD45 (30-F11, BioLegend, California, U.S.A.), and APC anti-mouse Ter119 (17-5921, eBioscience, San Diego, U.S.A.). The FACS plots showed that the surface markers of CD44, CD51, CD90, and CD105 were positive on MSCs, which was consistent with our previous reports [7,8,10]. MSCs were used for further experiments, when the CD45 negative Ter119 negative cells were up to 90%.

### Storage of MSCs

MSCs were suspended in CPDA-1 at a concentration of 5 × 10^6^/ml at 4 ± 2°C. The survival rate was tested on days 1, 4, 7, and 14 during storage through Trypan Blue (Mybiotech, A071) exclusion method. Meanwhile, the cells were stained with propidium iodide (PI, Sigma, P4170) to detect vitality on days 1 and 14. Flow cytometric data were acquired using FACS Calibur (BD Immunocytometry System, San Jose, U.S.A.) and analyzed with FlowJo software.

### RBCs quality assessment

RBCs quality assessment was performed in several aspects. RBC number, Hb and Hct levels were tested on Sysmex-100 instrument (Sysmex XP-300, Japan). Free Hb level was examined through free Hb kit (Nanjing Jiancheng Bioengineering Institute, A071). Lactate dehydrogenase (LDH) and potassium (K^+^)-iron levels were measured on biochemistry analyzer (Hitachi 7180, Japan). RBCs 2,3-diphosphoglycerate (2,3-DPG) was assessed by commercial 2,3-DPG kit according to the recommended protocols (AMEKO, mouse 2,3-DPG).

### Mouse model of acute anemia

A mouse model of acute anemia was established by intravenous injection of phenylhydrazine (PHZ, Sigma, 114715). Different concentrations (0.05, 0.10, and 0.15 mg/g of body weight) were examined to get an optimal condition. Fifty microliters of blood samples from mice were collected from eye vein and were suspended in tubes with 50 μl anticoagulant containing EDTA at different times, RBCs number, Hb and Hct levels were analyzed to evaluate anemia status [11]. The following experiments were carried out under the chosen PHZ concentration. Anemia assessment was expressed as the number of RBCs, Hb and Hct. The data were recorded to compare with ones after blood transfusion treatment.

The article "Mesenchymal stromal cells can be applied to red blood cells storage as a kind of cellular additive" was published in 2017. Journal: Biosci Rep.

### Statistical analysis

Statistical analyses were performed using Prism software v.6.1 (GraphPad). All data are presented as means ± S.D. Replications were done at least by three independent experiments. Results were analyzed with the unpaired Student’s *t*test, and *P*-value <0.05 was taken to indicate significance.

## Results

### MSCs reserved vitality in CPDA-1 medium

Although MSCs have been used both in experimental research and clinical research, how to reserve this multiple function cells was seldom touched. To determine the vitality of bone-associated MSCs maintained in CPDA-1 medium, we analyzed cells’ morphology and probed the survival. The result showed that MSCs were round and suspended without adherence, after 14-day storage in CPDA-1 medium at 4 ± 2°C (Figure 1A). When the viable cells were calculated after Trypan Blue staining, we found that the percentage of vital MSCs decreased along with the storage time, but more than 70.0% cells were still alive after 14 days (Figure 1B). The cells were further stained with PI to confirm this phenomenon. Flow cytometry analysis revealed that 75.3% living cells could be detected after 14-day storage (Figure 1C). These results suggested that MSCs stored in CPDA-1 buffer maintained their viabilities at least for 14 days at 4 ± 2°C.

**Figure 1:** The viability of MSCs reserved in CPDA-1 medium at 4 ± 2°C MSCs were suspended in CPDA-1 at 4 ± 2°C. (**A**) Photos of MSCs stained with Trypan Blue at the storage time for 1st and 14th days (upper line: magnification =10×, below line: magnification =20×). (**B**) The quantitative analyses of MSCs survival rate on the 1st, 4th, 7th, and 14th days during storage through Trypan Blue exclusion method. (**C**) FACS plot of the PI negative MSCs on 14th day. The red curve was unstained cells as the negative control. Data shown are from triplicate measurements.

### MSCs survived well and RBC vitality decreased at plateau

To evaluate the preservation of MSCs and RBCs at different sea levels, our detection was performed in local plain and plateau, respectively. We compared the alive MSCs between plain and plateau after storage for 14 days at 4 ± 2°C. The survival ratio of MSCs in plain region was 72.4%, while that in the plateau region was 70.6% (Figure 2A). When several independent measurements were integrated together, the data showed that there was no significant difference in the viability of MSCs between plain and plateau regions (Figure 2B). Meanwhile, we found that the number of RBCs significantly decreased at plateau region (Figure 2C); and the survival rates of RBCs were consistent with changes in RBCs number counts, which were also significantly decreased at plateau region (Figure 2D). Altogether, our data indicated that preservation at 2800 meters above sea level decreased the vitality of RBCs, while MSCs at the same high altitude underwent light damage.

The article "Mesenchymal stromal cells can be applied to red blood cells storage as a kind of cellular additive" was published in 2017. Journal: Biosci Rep.

**Figure 2:** The comparison of MSC or RBCs survival rates between plain and plateau MSCs and RBCs suspended in CPDA-1 at 4 ± 2°C were transported from plain to plateau. (**A**) FACS plot of the PI negative MSCs in plain and plateau. (**B**) Quantity of MSC survival rates between plain and plateau. (**C**) RBCs numbers between plain and plateau. (**D**) RBCs survival rates between plain and plateau. Data shown represent the mean ± S.D. from triplicate measurements.

### RBCs storage lesion was recovered by MSCs *in vitro*

Since MSCs maintained a good viability in CPDA-1 medium at plateau region, we were wondering whether MSCs could improve RBCs storage. Investigations were carried out under only RBCs standard preservation as control group accordingly. Experimental group of RBCs was stored together with MSCs (100:1). We found that the RBCs number count in experimental group was more than that in control group (Figure 3A). And the survival rate in experimental group was also higher than that in control group (Figure 3B). Numerous biochemical studies investigated RBCs’ metabolic modifications associated with the viability and the effectiveness [12–14]. RBCs hemolysis was the classical index of the storage effect of RBCs [4,15]. The data showed lesser free Hb was observed in RBCs stored with MSCs compared with that in the control group (Figure 3C). Both LDH and potassium levels in the supernatant decreased in RBCs stored with MSCs (Figure 3D,E), which was in consistence with free Hb changes. RBCs 2,3-DPG level is an important indicator of oxygen delivery. We found that the 2,3-DPG level increased significantly when RBCs were co-stored with MSCs compared with that of control group, implied that oxygen delivery could be improved (Figure 3F). Taken together, these results demonstrated that MSCs tended to recover RBCs storage lesion and maintain the viability and the effectiveness of RBCs.

The article "Mesenchymal stromal cells can be applied to red blood cells storage as a kind of cellular additive" was published in 2017. Journal: Biosci Rep.

**Figure 3:** The comparison of RBCs storage lesion between RBCs alone group and RBCs co-stored with MSC group at plateau RBCs with MSCs or not were preserved in CPDA-1 at 4 ± 2°C, which were transferred from plain to plateau for 10-day storage and returned to the plain. (**A**) The comparison of RBCs number counts. (**B**) The comparison of RBCs survival rates. (**C**–**F**) The supernatant of samples were tested for free Hb (C), LDH (D), K^+^ (E), and 2,3-DPG (F). Data shown represent the mean ± S.D. from more than three independent experiments.

### Murine anemia models were established

To determine the function of RBCs co-stored with MSCs *in vivo*, an anemia murine model should be established. The hemolytic activity of PHZ, may lead to acute hemolytic anemia in vertebrates [16]. First, we tried different concentrations of PHZ to inject the mice to get an applicable concentration. When the injection of PHZ was over 0.1 mg/g, the weight of mice obviously declined (Figure 4A). To test the anemia status, we analyzed RBCs number, Hb and Hct levels after injection of PHZ. RBCs number was the most decreased after the injection of 0.15 mg/g PHZ (Figure 4B). The levels of Hb and Hct were also the lowest after the injection of 0.15 mg/g PHZ (Figure 4C,D). The curves of RBC number, Hb and Hct levels showed that the artificial anemia maintained for 5 days (Figure 4B–D). When 0.15 mg/g PHZ were administrated into the mice for 1 day, RBCs counts, Hb and Hct levels were significantly decreased, which suggested that anemia model was successful (Figure 4E–G). Altogether, these data suggested that we established a successful anemia model by PHZ.

**Figure 4:** Murine anemia models were established by injection with PHZ (**A**) The weight of mice after injection different concentrations of PHZ. (**B**–**D**) The curves of RBCs number, Hb and Hct levels after injection with PHZ at different concentrations. (**E**–**G**) The comparisons of RBC number, Hb and Hct levels between control group and hemolysis group. The data were obtained from three independent experiments that included six mice per group.

### MSCs improved RBCs function on relieving anemia

After obtaining the anemia model, we further investigated RBCs function *in vivo* after co-storing with MSCs. All the RBCs were saved for 3 days in plain’s city, and then were transported to the plateau region. At plateau environment, RBCs were stored for another 10 days, and then transported to the original city. At 14th day, RBCs were transfused into anemic mice (Figure 5A). To confirm whether RBCs transfusion was successful, we set the CPDA-1 medium as the control group. We found a significant RBCs number increase after RBCs transfusion, compared with CPDA-1 medium transfusion (Figure 5B). Meanwhile, both Hb and Hct levels were elevated after RBCs transfusion (Figure 5C,D). These results demonstrated that RBCs transfusion was successful. After that, we also noticed the RBCs number was higher in co-stored group than that in RBCs group (Figure 5B). Both Hb and Hct levels in the co-stored group were also obviously higher, compared with that of RBCs group (Figure 5C,D). These results demonstrated RBCs that co-stored MSCs had a better effect on relieving anemia.

The article "Mesenchymal stromal cells can be applied to red blood cells storage as a kind of cellular additive" was published in 2017. Journal: Biosci Rep.

**Figure 5:** RBCs function *in vivo* after co-storing with MSCs (**A**) Experimental outline for data in (**B**–**D**). RBCs with MSCs or not were preserved in CPDA-1 for 3 days at plain. Then samples were transferred to plateau for 10-day storage and returned to the plain. At 14th day, samples were transfused into anemic mice through tail vein. After 24 h, the blood samples were collected from anemic mice by eye vein. (B–D) The comparisons of RBCs number, Hb and Hct levels from anemic mice transfused with RBCs amongst medium group, RBCs alone group, and RBCs co-stored with MSCs. The data were obtained from three independent experiments that included four mice per group.

## Discussion

In the present study, we first found MSCs preserved in CPDA-1 at 4 ± 2°C for 14 days still maintained great viability, even at plateau region. Meanwhile, we observed there were the storage lesions in RBCs in plateau during preservation, which was consistent with other studies [4]. Thus, we attempted to use MSCs as an available supplement to decrease RBCs lesion during storage. We found MSCs were helpful to support RBCs to maintain biochemical parameters and kept RBCs function well on relieving anemia. Thus, our findings provided a novel method of RBCs storage, which might be applied in human RBCs storage but still needed further exploration.

In the current research, we demonstrate MSC can remain vital within 14 days in CPDA-1 medium at 4 ± 2°C. Currently, liquid nitrogen storage and cell culture are two common methods for MSCs storage. However, liquid nitrogen storage at –196°C brings freezing impairment to cells. As for cell culture at 37°C in incubator, MSCs may undergo unpredictable differentiation. The method for MSCs storage used in our system is available, feasible, and simple, which may expand the useful prospects.

Recently, many clinical researches on the RBCs transfusion at different storage times have been reported [17–19]. How to store RBSs and the storage time are always the matter focussed by people. According to the function of MSCs on supporting RBCs to maintain biochemical parameters and relieving anemia, we believe that MSCs can be applied in RBCs storage as a kind of cellular additive. Numerous studies about RBCs storage strategies were designed to look for chemical components as additives [20–22]. A number of ASs are developed in the United States, including commercially available SAGM, MAP, PAGGGM, AS-1, AS-5 etc. which are all composed of varied chemical substrates [20,23,24]. Our research developed a novel concept to get a better storage effect for RBCs after cellular additive was administrated. In future, many cells may be found out whether they are suitable to improve the storage effect for RBCs. The storage effect for RBCs will be improved greatly, by adding chemical substrates and cellular additives.

The article "Mesenchymal stromal cells can be applied to red blood cells storage as a kind of cellular additive" was published in 2017. Journal: Biosci Rep.

We found RBCs storage lesion got worse, when RBCs were transferred from plain to plateau regions. So, it is an urgent need to seek the storage method of RBCs transfer. Our findings indicated that murine RBCs storage quality could be improved by co-storing with MSCs at the transfer process from plain to plateau regious, suggesting adding MSCs in preservation solution could be a new method to store RBCs, especially at the transfer process. If human RBCs storage quality could also be improved by adding MSCs in the preservation solution during the transfer process, it is helpful to keep the precious blood resource. Because there are some differences between human RBCs and murine RBCs, whether the storage of human RBCs could be improved by adding MSCs needs to be studied further.

However, some open questions still need further exploration. Our results did not include the therapeutic effect in anemic treatment using co-storing RBCs after 24 h. The long-term evaluation should be performed after transfusion *in vivo.* The mechanism why MSCs could improve RBCs storage, may light the facts that MSCs could affect cell microenvironment by the release of soluble factors or the transfer of cellular components to neighboring cells, in a way which significantly contributes to cell regulation [25,26]. But mechanistic studies about the specific role of MSCs in RBCs storage in more details are needed in future.

In summary, we found that MSCs could be preserved in CPDA-1 buffer at 4 ± 2°C, and demonstrated that MSCs were helpful to support RBCs to maintain biochemical parameters and keep RBCs functioning well in relieving anemia in mice models. Therefore, our observations suggested that MSCs may be used in RBCs storage as a kind of cellular additive.

## Abbreviations

AS: additive solution
CPDA-1: citrate phosphate dextrose adenine-1
Hb: hemoglobin
Hct: hematocrit
HSC: hematopoietic stem cell
LDH: lactate dehydrogenase
MSC: mesenchymal stromal cell
PHZ: phenylhydrazine
PI: propidium iodide
RBC: red blood cell
SAGM: saline adenine glucose mannitol
2,3-DPG: 2,3-diphosphoglycerate
